The article "Rare case of septic shock combined with meningitis caused by Pasteurella multocida without a history of cat and dog bites" was published in 2024. Journal: BMC Infect Dis.

# Rare case of septic shock combined with meningitis caused by *Pasteurella multocida* without a history of cat and dog bites

**DOI:** 10.1186/s12879-024-09207-1

**Published:** 2024-03-15

**Authors:** Yijun Zhu, Fang Zhu, Xiaoyun Shan, Jingchao Shi

**Affiliations:** 1 Department of Clinical Laboratory, Affiliated Jinhua Hospital, Zhejiang University School of Medicine, 321000 Jinhua, Zhejiang China; 2 Pathology Department, Affiliated Jinhua Hospital, Zhejiang University School of Medicine, 321000 Jinhua, Zhejiang China

**Keywords:** *Pasteurella multocida*, Bacteraemia, Sepsis, Septic shock, Meningitis

## Abstract

**Background:**

*Pasteurella multocida* is a zoonotic pathogen that mainly causes local skin and soft tissue infections in the human body through cat and dog bites. It rarely causes bacteraemia (or sepsis) and meningitis. We reported a case of septic shock and meningitis caused by *P. multocida* in a patient without a history of cat and dog bites.

**Case presentation:**

An 84-year-old male patient was urgently sent to the emergency department after he was found with unclear consciousness for 8 h, accompanied by limb tremors and urinary incontinence. In the subsequent examination, *P. multocida* was detected in the blood culture and wound secretion samples of the patient. However, it was not detected in the cerebrospinal fluid culture, but its DNA sequence was detected. Therefore, the patient was clearly diagnosed with septic shock and meningitis caused by *P. multocida*. The patient had no history of cat or dog contact or bite. The patient was subsequently treated with a combination of penicillin G, doxycycline, and ceftriaxone, and he was discharged after 35 days of hospitalisation.

**Conclusion:**

This report presented a rare case of septic shock and meningitis caused by *P. multocida*, which was not related to a cat or dog bite. Clinical doctors should consider *P. multocida* as a possible cause of sepsis or meningitis and should be aware of its potential seriousness even in the absence of animal bites.

## Background

*Pasteurella multocida* is a small Gram-negative, facultative anaerobic coccobacillus and one of the main zoonotic pathogens; it is present in the oral cavity and gastrointestinal tract of many domestic animals, wildlife, and birds [1]. The highest colonisation rate is found in cats (50–90%), followed by dogs (55–60%), pigs (51%), and rats (14%) [2]. This bacterium is mainly transmitted through scratches and bites from animals such as cats and dogs, causing local skin and soft tissue infections in humans. Reports have also documented transmission through non-traumatic routes, including inhalation of aerosols contaminated by pet waste or transmission from pet secretions such as saliva, leading to pneumonia [3]. *P. multocida* can also cause severe systemic infections, such as bacteraemia, sepsis, septic shock, peritonitis, and meningitis, but these infections are extremely rare. A 14-year study in France found that only 14 of 215 cases of *P. multocida* infections were bloodstream infections, accounting for 6.5% of the total infections [4]. Another study has shown that the mortality rate of patients with *P. multocida* bacteraemia is between 14% and 31% [5]. In August 2022 we treated a case of *P. multocida* septic shock combined with meningitis in a patient without a history of cat or dog bites.

The article "Rare case of septic shock combined with meningitis caused by Pasteurella multocida without a history of cat and dog bites" was published in 2024. Journal: BMC Infect Dis.

## Case presentation

On day 0, an 84-year-old male patient was sent to the emergency department after he was found with unclear consciousness for 8 h, accompanied by limb tremors and urinary incontinence. His blood pressure was 78/53 mmHg, and his temperature was 38.4 °C. The blood test showed the following: white blood cell count of 6.57 × 10^9^ /L, with 90.6% neutrophils; haemoglobin level of 111 g/L; red blood cell count of 3.19 × 10^12^ /L; and platelet count of 72 × 10^9^ /L. His procalcitonin level was 14.84 ng/mL (reference value: 0–0.06 ng/mL; >2.0 ng/mL, high risk of infection), interleukin-6 was > 50,000 pg/mL (reference value: 0–10 pg/mL), and D-dimer was 10,349 µg/L (reference value: <500 µg/L). His COVID-19 nucleic acid test was negative. Blood gas analysis revealed the following: potassium ion level of 2.70 mmol/L, sodium ion level of 133.0 mmol/L, actual bicarbonate level of 16.0 mmol/L, total carbon dioxide level of 14.5 mmol/L, base excess of -6.9 mmol/L, oxygen saturation of 98.8%, and lactate level of 8.3 mmol/L. Head CT showed postoperative changes in the right side of the skull, subdural haematoma on the left frontal and parietal regions, and slight bleeding on the right frontal lobe. After being diagnosed by doctors in the intensive care unit (ICU), the patient was initially diagnosed with shock and intracranial infection, and he was subsequently sent to the ICU for further treatment.

On day 0, physical examination after admission showed that the patient was in a coma with a body temperature of 36.8 °C, a pulse rate of 91 beats per minute, a respiratory rate of 28 times per minute, and a blood pressure of 69/38 mmHg. The patient’s neck was soft and had no resistance. The breath sounds in both lungs were coarse, the heart rhythm was regular, no pathological murmurs were heard in the valve area, and a slight wheezing sound was observed. The lower limbs had no oedema, but an unhealed wound was found on the left lower limb (Fig. 1). The Babinski sign was negative in both lower limbs. The patient had a history of hypertension (irregular treatment), appendectomy, craniocerebral trauma surgery (twenty years ago), hernia surgery, and measles.

The article "Rare case of septic shock combined with meningitis caused by Pasteurella multocida without a history of cat and dog bites" was published in 2024. Journal: BMC Infect Dis.

**Fig. 1:** Wound with broken skin on the lower left limb

Further examinations were conducted, and the patient’s family was informed of his critical condition. Symptomatic treatments such as fluid replacement, gastric protection, expectorant therapy, and blood transfusions were administered. Because of the possibility of intracranial infection, the patient was empirically treated with meropenem for anti-infection.

On day 1, the Microbiology Laboratory reported a critical value: four blood culture bottles (anaerobic and aerobic bottles) sent for examination on day 0 were all positive for *P. multocida* (Figs. 2, 3 and 4). The patient’s wound secretions were collected for bacterial culture.

**Fig. 2:** Isolated strain of *P. multocida* on sheep blood plates,The formed colonies are opaque, light-grey. (cultured at 35 °C for 24 h)

**Fig. 3:** *P. multocida* is a short Gram-negative rod or coccobacillus (Gram staining, ×1000)

**Fig. 4:** Mass spectrometry identification of *P. multocida*

On day 3, the drug sensitivity test results for this bacterial species were reported: sensitive to penicillin G, ampicillin, amoxicillin/clavulanic acid, ceftriaxone, levofloxacin, trimethoprim/sulfamethoxazole, chloramphenicol, and tetracycline but resistant to erythromycin. After consultation with the Infectious Disease Department, the patient was treated with penicillin G(3.2 million units, intravenous drip every 4 h) and doxycycline (100 mg every 12 h, oral administration, with an initial dose of 200 mg) for anti-infection. The CSF examination showed white blood cells at 6495/µL, neutrophil ratio at 95%, LDH at 377 U/L (reference value: <40 U/L), glucose at < 1.1 mmol/L (reference value: 2.2–3.9 mmol/L), protein at > 6000 mg/L (reference value: 120–600 mg/L), and chloride at 120.9 mmol/L (reference value: 120–130 mmol/L). The CSF specimen was negative for bacterial culture, but next-generation gene sequencing (NGS) detected *P. multocida* (DNA sequence number: 14,235), confirming a diagnosis of bacterial meningitis. Therefore, the anti-infection treatment was changed to ceftriaxone sodium (2 g, intravenous drip, once every 12 h; Table 1).

**Table 1:** Timeline of the patient’s diagnosis and treatment

Date	Time	Events
Day 0	Morning	The patient experienced sudden illness, fell, and subsequently lapsed into a coma.
	12:31	The patient was taken to the emergency room.
	13:05	Blood samples were collected for blood culture (bilateral double bottle).
	13:12	Head CT examination was performed.
	13:52	Imipenem was intravenously infused as empirical medication.
	17:46	The patient was transferred to the ICU.
	19:11	Meropenem was intravenously infused as empirical medication.
Day 1	9:56	Intravenous meropenem infusion was continued as empirical medication.
	10:03	Wound secretions were collected for bacterial culture.
	10:43	According to the clinical microbiology laboratory report, four blood culture bottles tested positive for Gram-negative bacteria.
	14:33	According to the clinical microbiology laboratory report, *P. multocida* was present in the blood culture samples.
	16:32	The initial dose of penicillin G 3.2 million units + 0.2 g oral doxycycline was administered.
Day 2	2:01	The subsequent dose of penicillin G 3.2 million units + 0.1 g oral doxycycline was administered.
	8:00	CSF was collected for bacterial culture and NGS detection.
	Evening	The NGS results of CSF revealed 14,235 sequences of *P. multocida* genes.
Day 3	7:50	Intravenous infusion of 2 g of ceftriaxone sodium was initiated.
	8:52	The clinical microbiology laboratory released the drug sensitivity results of *P. multocida*.
	12:14	The patient underwent CSF replacement.
	16:37	Intravenous drip of 2 g of ceftriaxone sodium was continued.
Day 4	17:00	The clinical microbiology laboratory revealed the drug sensitivity results of *P. multocida* cultured from the patient’s wound secretions.
Day 5	9:38	The clinical microbiology laboratory detected no pathogenic bacteria in the CSF after 3 days of cultivation.

CT: Computed Tomography; ICU:Intensive Care Unit; CSF:Cerebrospinal Fluid; NGS:Next-generation Gene Sequencing

On day 4, *P. multocida* was detected in the wound secretion on the left lower limb. The drug sensitivity results were consistent with the bacteria isolated from the blood culture. A lumbar puncture was also performed for CSF replacement.

The article "Rare case of septic shock combined with meningitis caused by Pasteurella multocida without a history of cat and dog bites" was published in 2024. Journal: BMC Infect Dis.

After more than 20 days of anti-infection treatment, the patient’s condition gradually improved. On day 29, when stable vital signs were recorded, the tracheal intubation was removed. Finally, the patient was discharged after 35 days of hospitalisation.

## Discussion and conclusion

*P. multocida* was named after Louis Pasteur, who first described the bacterium as a pathogenic factor for poultry cholera in 1881 [6]. The first human infection was reported in 1914. This bacterium mainly exists in the mouth and throat of healthy animals, especially cats, dogs, and pigs, as well as various wild animals [7]. Its positive rate in poultry in Jiangxi Province, China is 6.39% (14/219) [8]. This pathogenic bacterial species infects humans through scratching, biting, licking, kissing, and sharing food with pets [6]; vertical transmission from pregnant women to foetuses has also been reported [9].

Infections caused by *P. multocida* can be divided into three types [10]. The most common type is infection caused by animal bites and scratches, mainly leading to local skin and soft tissue infections [11]. The second type is respiratory tract infection, which includes pneumonia, empyema, and lung abscess. The third type includes other systemic infections, such as bacteraemia, endocarditis, meningitis, brain abscess, spontaneous bacterial peritonitis, and abdominal abscess [7]. A 20-year study in Australia found that the crude incidence of *Pasteurella* spp. infections increased from 1.5 per 100,000 population in 2000 to 11.4 per 100,000 population in 2021. It also revealed 22 (11.3%) bloodstream infections, 22 (11.3%) invasive infections, 34 (17.4%) deep local infections, 98 (50.2%) superficial infections, and 19 (9.7%) other or unknown infections [12]. The susceptibility factors of *Pasteurella* sepsis include underlying diseases such as diabetes, liver cirrhosis, chronic obstructive pulmonary disease, hypertension, malignant tumours, immunodeficiency, and advanced age [11, 13].

The patient in this case was an 84-year-old widowed elderly person who does not keep cats, dogs, or other pets and has no history of being bitten by them. However, he keeps chickens, ducks, and other poultry at home and has had close contact with them. Whilst working in the fields, he had an abrasion on the lower limbs that developed into a wound. He had a close contact with the poultry whilst caring for them. We speculated that the oral cavity of poultry might have carried *P. multocida*, which infected patients through their wounds. Because of his underlying conditions such as hypertension and old age, his immune function was poor, and *P. multocida* that entered the body caused sepsis and meningitis. Microbial examination results also showed that the wound secretions and blood cultures had *P. multocida* growth. Although this bacterial species was not detected in the CSF culture, NGS detected 14,235 DNA sequences of *P. multocida*. Its DNA remained even though the antibiotics used before CSF sample collection eradicated the bacteria in the CSF.When the patient was admitted, he had high levels of inflammatory markers such as neutrophils, procalcitonin, and interleukin-6, accompanied by hypotension, multiple organ failure, and intracranial infection symptoms such as confusion and convulsion. Clinical and laboratory examinations supported the diagnosis of septic shock combined with meningitis caused by *P. multocida*.

Currently, no guidelines or expert consensus has been reached for the treatment of bacteraemia caused by *P. multocida* [7]. This bacterium is generally sensitive to penicillin, which is used as the first-line treatment. However, a case report indicated that *P. multocida* can produce beta-lactamases, resulting in penicillin resistance [14]. In such rare cases, second- or third-generation cephalosporins, fluoroquinolones, or tetracyclines can be used. Other cases revealed that *P. multocida* bacteraemia can also be successfully treated using various antibiotics such as piperacillin/tazobactam, aztreonam [15], ceftriaxone combined with ampicillin [16], cefepime, and amoxicillin/clavulanic acid. Macrolides are not recommended because of their high resistance rates and unpredictable sensitivity [17]. *P. multocida* isolated from different hosts and regions may exhibit multiple drug resistance to various antibiotics [18], which may be related to the widespread use of such antibiotics in animal feed. Antibiotic susceptibility results revealed that it was sensitive to penicillin, ampicillin, amoxicillin/clavulanic acid, ceftriaxone, levofloxacin, trimethoprim/sulfamethoxazole, chloramphenicol, and tetracycline, but it was resistant to erythromycin. After obtaining the blood culture results, we treated the infection with penicillin G and tetracycline. The positive CSF result indicated that the patient had concurrent *P. multocida* sepsis and meningitis. Therefore, the anti-infection treatment was changed to ceftriaxone, an antibiotic with superior blood–brain barrier permeability. After a 25-day treatment, the follow-up blood culture was negative; the patient gradually recovered and was finally discharged.

The article "Rare case of septic shock combined with meningitis caused by Pasteurella multocida without a history of cat and dog bites" was published in 2024. Journal: BMC Infect Dis.

*P. multocida* can lead to complications such as purple fingertips [19], purpura fulminans [20], peritonitis [21], pyosalpinx [22], mycotic aneurysm [23], meningitis, and endocarditis. Non-bite patients are more likely to develop bacteraemia [7], and such bacteraemia is more severe that it requires ICU treatment. Infections related to non-animal bites mainly occur in patients with severe complications and immunodeficiency, which can easily lead to systemic infections. Patients with non-bite bacteraemia require ICU treatment, have longer hospital stays, and have high mortality rates. Therefore, active treatment measures for immunocompromised patients should be taken [7].

*P. multocida* grows well on blood agar and chocolate agar, but it does not generally grow on MacConkey agar [24]. After 24 h of cultivation at 35 °C, it forms opaque, light-grey colonies with a diameter of 1–2 mm on blood plates, which are similar to those of *Staphylococcus epidermidis* and can be identified by Gram staining. In sputum cultures, *P. multocida* may be missed because of the overgrowth of normal oral flora on agar. In addition, the identification of *P. multocida* using a VITEK-2 bacterial identification system is unsatisfactory [25]. Nevertheless, *P. multocida* can be accurately identified by 16 S rRNA sequencing or MALDI-TOF mass spectrometry [26]. In the present case, the isolated strain from this patient was rapidly identified using a MALDI-TOF mass spectrometer. Drug sensitivity was tested using the VITEK-Compact2 microbial identification and drug sensitivity system. The breakpoint for the drug sensitivity test was determined according to the standards established by the Clinical and Laboratory Standards Institute (CLSI) in 2021. The drug sensitivity test served as a basis for a clinical anti-infection treatment. With improvements in the quality control system, the NGS technology has been widely used to detect pathogens in various clinical specimens [27]. Q-mNGS ™ 2.0 technology was applied to detect pathogenic DNA in the patient’s CSF. This technology is based on an Illumina sequencing platform and PCR-free library construction technology. The proportion of human nucleic acids and the content of pathogenic microorganisms in the samples are quantitatively detected by adding artificially synthesised tag sequences to the samples. The host index, which reflects the content of nucleic acids in humans, and the Q-index, which reflects the level of pathogenic microorganisms, can be directly compared between different specimens. Q-mNGS ™ 2.0 technology was successfully used to detect the DNA of *P. multocida* in the patient’s CSF. Thus, it provided a basis for the diagnosis of meningitis.

The article "Rare case of septic shock combined with meningitis caused by Pasteurella multocida without a history of cat and dog bites" was published in 2024. Journal: BMC Infect Dis.

In summary, this case report described a rare case of septic shock and meningitis caused by *P. multocida* in a patient without a history of cat or dog bites. This finding suggested that clinical doctors should consider *P. multocida* as a potential cause of sepsis or meningitis and be aware of its potential severity even in the absence of animal bites. Furthermore, individuals should protect their wounds as much as possible in daily life and prevent wounds from coming into contact with poultry or pets.

## Data Availability

The datasets used and/or analysed during the current study available from the corresponding author on reasonable request.

## Abbreviations

COVID-19: Corona Virus Disease 2019
CT: Computed Tomography
ICU: Intensive Care Unit
CSF: Cerebrospinal Fluid
LDH: Lactate Dehydrogenase
NGS: Next-generation Gene Sequencing
DNA: Deoxyribonucleic acid
rRNA: ribosomal Ribonucleic Acid
MALDI-TOF: Matrix-Assisted Laser Desorption/ Ionization Time of Flight

## References

[1] Samarkos M, Fanourgiakis P, Nemtzas I (2010). Pasteurella multocida bacteremia, spontaneous bacterial peritonitis and septic arthritis in a cirrhotic patient. Hippokratia.

The article "Rare case of septic shock combined with meningitis caused by Pasteurella multocida without a history of cat and dog bites" was published in 2024. Journal: BMC Infect Dis.

[2] Miyoshi S, Hamada H, Miyoshi A (2012). Pasteurella multocida pneumonia: zoonotic transmission confirmed by molecular epidemiological analysis. Geriatr Gerontol Int.

[3] Cabras O, Turmel JM, Olive C (2022). COVID-19 and Pasteurella multocida Pulmonary Coinfection: a Case Series. Trop Med Infect Dis.

[4] Dernoncourt A, Lacroix M, Duhaut P (2022). Prognostic factors of Pasteurella infections: a single-center retrospective cohort study over a 14-year period (2005–2018). Int J Infect Dis.

[5] Chatelier E, Mahieu R, Hamel JF (2020). Pasteurella bacteraemia: impact of comorbidities on outcome, based on a case series and literature review. Int J Infect Dis.

[6] Kukrety S, Parekh J, Townley T (2016). Pasteurella multocida Bacteremia in an immunocompromised patient. Case Rep Med.

[7] Giordano A, Dincman T, Clyburn BE (2015). Clinical features and outcomes of Pasteurella multocida infection. Med (Baltim).

[8] Tan MF, Li HQ, Yang Q (2023). Prevalence and antimicrobial resistance profile of bacterial pathogens isolated from poultry in Jiangxi Province, China from 2020 to 2022. Poult Sci.

[9] Scheurer JM, Fanta ML, Colbenson GA (2022). Early-Onset neonatal Sepsis caused by Vertical Transmission of Pasteurella multocida. AJP Rep.

[10] Weber DJ, Wolfson JS, Swartz MN (1984). Pasteurella multocida infections. Report of 34 cases and review of the literature. Med (Baltim).

[11] Aljameely A, Wali G (2019). Pasteurella multocida septic shock: Case Report and Literature Review. Case Rep Infect Dis.

[12] Mahony M, Menouhos D, Hennessy J (2023). Spectrum of human Pasteurella species infections in tropical Australia. PLoS ONE.

[13] Nollet V, Souply L, Rosolen B (2016). Risk factors for invasive pasteurellosis: a retrospective case study. Eur J Clin Microbiol Infect Dis.

[14] Naas T, Benaoudia F, Lebrun L (2001). Molecular identification of TEM-1 beta-lactamase in a Pasteurella multocida isolate of human origin. Eur J Clin Microbiol Infect Dis.

[15] Winner JS, Gentry CA, Machado LJ (2003). Aztreonam treatment of Pasteurella multocida cellulitis and bacteremia. Ann Pharmacother.

[16] Clarke DA, Mcbride A, Kelsey M (2017). Pasteurella multocida meningoencephalitis in an immunocompetent adult with multiple cat scratches. BMJ Case Rep.

[17] Ferreira J, Treger K, Busey K (2015). Pneumonia and disseminated bacteremia with Pasteurella multocida in the immune competent host: a case report and a review of the literature. Respir Med Case Rep.

[18] Zhang R, Tian S, Zhang T (2023). Antibacterial activity mechanism of coptisine against Pasteurella multocida. Front Cell Infect Microbiol.

The article "Rare case of septic shock combined with meningitis caused by Pasteurella multocida without a history of cat and dog bites" was published in 2024. Journal: BMC Infect Dis.

[19] Zarlasht F, Khan M (2018). A case of recurrent Pasteurella bacteremia in an Immunocompetent patient with no animal bite. Am J Case Rep.

[20] Fukuhara A, Fushimi S, Nakata M (2023). Venoarterial extracorporeal membrane oxygenation treatment for acute respiratory distress syndrome and non-occlusive mesenteric ischemia due to Pasteurella multocida-related sepsis with purpura fulminans: a case report. Int J Emerg Med.

[21] Mohan P, Diaz AR, Lee S (2023). Pasteurella multocida bacteremia: a case report of pelvic cavity inflammation with abnormal uterine bleeding, fever, and sclerotic bone lesions. IDCases.

[22] Myckan KA, Booth CM, Mocarski E (2005). Pasteurella multocida bacteremia and tuboovarian abscess. Obstet Gynecol.

[23] Orgiu A, Zanier T, Kashi-Dakhil M (2020). An unusual presentation of mycotic popliteal artery pseudoaneurysm due to Pasteurella multocida infection. Int J Angiol.

[24] Desem MI, Handharyani E, Setiyono A (2023). Morphology, biochemical, and molecular characterization of Pasteurella multocida Causing Hemorrhagic Septicemia in Indonesia. Vet Med Int.

[25] Guillard T, Duval V, Jobart R (2009). Dog bite wound infection by Pasteurella dagmatis misidentified as Pasteurella pneumotropica by automated system Vitek 2. Diagn Microbiol Infect Dis.

[26] Zangenah S, Güleryüz G, Boräng S (2013). Identification of clinical Pasteurella isolates by MALDI-TOF - - a comparison with VITEK 2 and conventional microbiological methods. Diagn Microbiol Infect Dis.

[27] Schlaberg R, Chiu CY, Miller S (2017). Validation of Metagenomic Next-Generation sequencing tests for Universal Pathogen Detection. Arch Pathol Lab Med.

